RETRACTED

# Discussion on Protein Metabolism and Requirement of Aerobics Athletes during Training Based on Multisensor Data Fusion

**DOI:** 10.1155/2022/6169150

**Published:** 2022-03-12

**Authors:** Hua Gong, Shuang Chen, Shuo Yu, Dong Liu, Xin Li, Zeliang Shan, Fan Kong, Zhi Yan, Feng Han

**Affiliations:** ^1^Liaoning Normal University Sports Institute, Dalian 116029, Liaoning, China; ^2^Department of Medical Health, Xing'an Vocational and Technical College, Ulanhot 137400, Inner Mongolia, China; ^3^Sports Department of Liaoning Agricultural Technical College, Yingkou 115009, Liaoning, China; ^4^Health College, Polus International College, Chengdu 610103, Sichuan, China; ^5^Physical Education Department, Luxun Academy of Fine Arts, Dalian 116029, Liaoning, China; ^6^Rehabilitation and Nursing Institute, Tianfu College of Swufe, Chengdu 610103, Sichuan, China; ^7^School of Physical Education and Health, Dalian University of Technlogy, Dalian 116029, Liaoning, China; ^8^Orthopaedics, Dalian Port Hospital, Dalian 116001, Liaoning, China

## Abstract

Competitive aerobics has emerged as a highly competitive sport beyond its own physical limit. Modern competitive aerobics competition is very fierce; athletes cannot only rely on a specific competitive skill to achieve good results. Protein is the physical basis of life activity. The life activity of human body is closely related to protein, and protein is closely related to human exercise ability. This article aims to study protein metabolism and demand of aerobics athletes during training based on multisensor data fusion. A total of 26 female aerobics athletes were randomly divided into two groups: exercise group and exercise + nutrition group. According to the characteristics of human motion, a comprehensive measurement acquisition sensor system for collecting human motion information is designed and implemented, and the system is used to monitor the subject's protein condition in real time. The subjects took protein nutrient solution before breakfast every day. The dynamic recognition algorithm designed in this paper also has shortcomings, and the monitoring protein method based on gait and other signs is not completely correct. The experiment lasted for 7 weeks. The results showed that the level of serum transferrin receptor decreased significantly in the quiet + nutrition group for 4 weeks, which was significantly different from that at 0 and 3 weeks in the same group (*P* < 0.01) and was significantly different from that in the same group at 7 weeks (*P* < 0.05). In the exercise group, the level of serum transferrin receptor increased significantly at 5 weeks, compared with the same group at 0 and 3 weeks (*P* < 0.05).

RETRACTED

## 1. Introduction

The technical level of competitive aerobics is affected by factors such as physical quality, psychological quality, technical ability, sense of music, and expressiveness of athletes. The development of computer technology can be used for the daily training of competitive gymnastics, so the aerobics technology of athletes can use advanced computer technology. When aerobics athletes fail to exercise for a long time, protein can provide energy up to 5%–18% of the total exercise energy consumption. Exercise can make the human body protein metabolism change, but different nature of the exercise produced different effects, so protein requirements for athletes at different events are not the same. Accurately identifying the athlete's protein condition can accurately understand the physical condition and improve the target point and realize the personalized and precise supplement of the athlete. Nanopore sensing technology can detect protein changes from a single-molecule level, effectively improving the accuracy of detecting athletes' protein conditions. This topic uses nanopore single-molecule sensors to carry out experimental studies on single-protein molecules and protein interaction relationships.

The effect of exercise on lipoprotein metabolism has been studied for many years. Although there are some differences in the results due to different exercise modes, intensity, and research objects, a large number of epidemiological and clinical investigations have confirmed the following: No matter for men, women, old people, or children, China-Africa daily health life habits and lack of exercise or low fitness levels and many cardiovascular disease risk factors and incidence of coronary heart disease (CHD) were positively correlated, while regular exercise can effectively reduce blood lipids and lipoproteins and make the original plasma lipoprotein atherosclerosis develop in a good direction, and at the same time, it can control and reduce the risk factors of cardiovascular disease or coronary heart disease and slow down the adverse effects of aging [1, 2]. In order for the human body to exercise normally, the human body needs to consume more protein energy and supplementary food to promote the normal operation of the body.

Some scholars asked 166 athletes to maintain a scientific diet for three consecutive days, train more than 3 hectares of specific physical activities per week, and then be converted into macronutrients by a nutritionist. During Goodyear and other snow and ice athletes' training, the daily protein requirements were as follows: when the training amount was small, male speed skating athletes were 139 g/d and female athletes were 95 g/d. Skiing events male athletes were 110 g/d and female athletes were 64 g/d. When the training volume is large, the speed skaters are 165 g/d for men and 106 g/d for women [3]. At the same time, it is suggested that when the amount of exercise increases, the urine nitrogen excretion of athletes increases, and the nutrition level of protein can be understood by hemoglobin measurement. Crouse et al. found that the local levels of insulin and amino acids in muscles play an important role in controlling the synthesis of myostatin, and the reduction of insulin secretion caused by hunger reduces the synthesis rate of skeletal muscle protein by more than 50%, which is related to inhibiting the initiation of protein synthesis [4].

RETRACTED

The innovation of this paper is the use of sensors to monitor protein changes in gymnasts, enabling visualization of athletes' protein requirements. At present, because calisthenics is very important to the development of students' physical quality, major universities widely carry out this sport. The aerobics center of each province will bring some aerobics trainers to participate in the intensive training, so that they will be fully prepared for the higher level of competition, as a professional aerobics athlete to achieve outstanding results. Aerobics athletes' training is not only the most basic technical movement training but also physical training. The results showed that the serum transferrin receptor level in the quiet + nutrition group decreased significantly after 4 weeks, which was significantly different from that of the same group at 0 weeks and 3 weeks (*P* < 0.01) and significantly different from that of the same group at 7 weeks (*P* < 0.05). In the exercise group, the serum transferrin receptor level was significantly increased at week 5, which was significantly different from that of the same group at weeks 0 and 3 (*P* < 0.05), showing that the serum transferrin receptor level at weeks 0 and 3 was significantly lower than that at week 5.

## 2. Protein Demand and Monitoring

### 2.1. Physiological Functions of Proteins

Human life is inseparable from proteins, which are an important part of human cells. Proteins have different structures and have many physiological functions. Their main functions are as follows.

#### 2.1.1. Catalytic Function

In order to maintain the balance of human functions, the human body needs to produce some chemical reactions. Enzyme is a catalyst, and many chemical reactions are completed under the action of enzymes, so it can effectively control the metabolism of the human body and expel wastes from the body. According to scientific testing, the main components of the human body are more than 1,000 kinds of enzymes and proteins. Proteins have certain catalytic functions, so they are important substances to maintain human body functions [5].

RETRACTED

#### 2.1.2. Transportation Function

The human body is an organic whole, and blood circulation and oxygen transport need carriers. Protein is an effective carrier and an effective tool to ensure the normal transport of the human body. Effective transport of human body functions requires its normal operation to effectively complete its transport and guarantee its organic circulation [6].

#### 2.1.3. Motor Function

The movement of the human body mainly relies on muscles to complete, and protein is the main component of muscles. There is a certain relationship between muscle contraction and relaxation and protein quality. The muscles of athletes are usually more developed than our ordinary people because athletes have a certain standard of diet, and there are requirements for daily intake of protein, fat, water, and so on [7, 8].

#### 2.1.4. Hormone Function

In biology, the main component of many hormones is protein, which has a certain therapeutic effect on patients in medicine. Protein and polypeptide hormones are important hormones in animals, which regulate and control the physiological activities of animals. For example, insulin can reduce blood sugar. Glucagon has 3485 polypeptides of 29 amino acid residues. Its effect is exactly opposite to that of insulin, which can promote glycogen decomposition and gluconeogenesis and increase blood glucose concentration. Hormones are often available in people's lives, but the use of hormones should be reduced to a certain extent to cause damage to the human body. Proteins have certain hormonal functions and are the main components of hormones [9]. The flow chart of physiological function of protein is shown in Figure 1.

### 2.2. Function of Protein during Exercise

1. Protein is the basic structure of cells. Protein is the main component of cells, accounting for more than 80% of the dry weight of cells; proteins constitute the cell membrane and intracellular materials and regulate genetic information. The tissue cells of the body are in a balance of constant aging and renewal, and protein is the raw material for maintaining tissue repair and regeneration. Physical exercise can strengthen the metabolism of the human body. Therefore, it can strengthen the bones and muscles and increase the content of protein in the body [10].
2. Proteins have physiological functions of regulating the body. All biochemical reactions in the body require the participation of enzymes with catalytic activity (with very few exceptions), and enzymes are essentially proteins. Proteins play an important role in regulating the acid-base balance of body fluids. When intense exercise leads to the enhancement of enzyme metabolism, blood proteins play an important role in buffering, thus keeping the internal environment of the body relatively stable. Many of the hormones regulating human physiological functions are composed of compounds of different amino acids and proteins, such as insulin and pituitary hormones regulating blood glucose levels [11].
3. Proteins participate in energy supply during exercise. During long and intensive exercise, proteins, especially the free amino acids in the human body, can also participate in energy supply as energy materials, but the overall participation ratio is not high, generally accounting for 5%–18% of the total energy consumption. Amino acids derived from tissue protein regeneration also contribute a certain amount of energy. However, in exercise, protein takes a relatively small proportion in energy supply. Only when the body consumes insufficient sugar and fat in the body does the body break down protein to produce amino acids and obtain energy [12].

RETRACTED

### 2.3. Effects of Exercise on Protein Metabolism

#### 2.3.1. The Influence of Strength Training on Protein Metabolism

The athlete receives the strength movement training for a long time, can promote the protein anabolism obviously, and increases the muscle strength and the volume. Strength training makes the volume of training muscle increase, muscle fiber thicken, and strength enhanced. This adaptation occurs in fast-twitch muscle fibers. The main reason for muscle enlargement is the increase of muscle protein, including the increase of contractile protein. In addition, the amount and strength of connective tissue, tendons, and ligaments surrounding muscle fibers also increase.

Strength training can stimulate insulin secretion; for example, centripetal movement training can increase the sensitivity of muscle cells to insulin stimulation. Centrifugal exercise reduced the sensitivity of muscle cells to insulin stimulation, and this reduction lasted for more than two days after exercise. Metabolic studies have shown that this change is related to the reduction of the glucose transport rate by centrifugal motion, which leads to the slowdown of the glycogen synthesis rate. The sensor designed in this paper observes this feature and completes the monitoring task based on this principle. This temporary insulin resistance and inhibition of glycogen regeneration can lead to hyperinsulinemia, which may increase the rate of myoprotein synthesis.

#### 2.3.2. The Influence of Endurance Training on Protein Metabolism

Endurance training increased the number and volume of mitochondria, as well as the activity of mitochondrial proteins and constituent enzymes. During endurance exercise, arginine stimulates insulin secretion. Aerobic exercise inhibits insulin secretion, increases insulin receptor sensitivity, and improves glucose tolerance. The effect of this movement also affects the metabolism of the body during the quiet state, so that the fluctuation frequency of insulin secretion remains unchanged, while the amount of insulin secretion decreases at each peak. Insulin and amino acids play an important role in controlling the synthesis of muscle protein in local muscles. Reduced insulin secretion caused by starvation reduced the rate of skeletal muscle protein synthesis in animals by more than 50%. The mechanism is related to inhibiting the initiation of protein synthesis and involves the phosphorylation of the translation regulator eukaryotic promoter 4E (EIF-4E) binding protein 1 (4E-BP1). In this process, insulin-like growth factor I (IGF-I) promotes phosphorylation of 4E-BP1 and dissociation of the 4E-Bp1-EIF-4E complex, promoting protein synthesis. Therefore, the decrease of insulin level caused by endurance exercise is one of the mechanisms controlling muscle protein synthesis. This is reflected in the difference of muscle mass between endurance athletes and strength athletes and also reflects the physiological adaptation mechanism of the body to meet the needs of different forms of exercise.

RETRACTED

### 2.4. Endurance Exercise and Protein Metabolism

When the human body carries out physical exercise, the proportion of protein energy supply is generally small, accounting for about 5%–7% of the total thermal energy needs. However, with the gradual depletion of glycogen in exercise, the proportion of protein energy supply also increases correspondingly, and the maximum can rise to about 15% of the total thermal energy needs. It can be seen that the main exercise type that has great influence on protein metabolism is endurance exercise.

During prolonged endurance exercise, the limited sugar reserves in the body are consumed in large quantities and the gluconeogenic pathway of amino acids is activated. After the removal of amino acids, most of the carbon skeleton in the body can enter the tricarboxylic acid cycle or glycolytic metabolism pathway. After oxidation, energy is generated, which can also be converted into glucose to help maintain blood sugar concentration. Among them, alanine and glutamine accounted for about 30% of amino acid isoglucose. In the process of body movement, pyruvate produced by myoglycogen oxidation reacts with amino acids such as lysine to form alanine. In this step, the amino acids that provide amino acids are converted to ketoacids, which enter the aerobic metabolic pathway for oxidative energy supply. The generated alanine enters the blood and is transported to the liver, where it is regenerated into glucose through the glucogenic metabolic pathway of the liver, so as to increase the source of blood glucose in exercise, so it is called alanine glucose circulation. The glucose-generating process of glutamine also has a similar glutamine-glucose cycle.

RETRACTED

### 2.5. The Protein Requirement of Athletes

The diet of athletes must have scientific standards. The protein intake of athletes has a certain relationship with sports, weight, and so on. The same sports, different genders, different weights, and different training intensities have certain standards for protein intake. A nutritionist needs to make a reasonable diet according to the actual situation of the athlete to promote the healthy growth of the athlete. Studies have shown that the daily protein requirement of long-term moderate intensity exercise is 2.5–3.0 /kg body weight. The daily protein requirement of athletes in bunker weight and speed and strength events is 2.4–2.59/kg body weight. The protein requirement of athletes is a general standard, and there are certain differences in the research data of experts and scholars in different industries. Strictly speaking, different athletes have certain differences in protein requirements. Nutritionists need to consume protein reasonably according to the physical condition of athletes, scientifically adjust the physical functions of athletes, and maximize their training effects.

### 2.6. The Relationship between Protein Metabolism and Exercise

#### 2.6.1. Protein Synthesis

Protein cooperation is related to the intensity of exercise; the greater the intensity of exercise, the slower the protein synthesis. In animal experiments, a fast-running mouse made protein about 70 percent slower than a normal mouse. Therefore, there is a certain relationship between protein metabolism and sports. Athletes synthesize protein more slowly than ordinary people, which plays a certain role in protein maintenance of body functions. Therefore, scientific data must be used to illustrate the relationship between protein and sports.

#### 2.6.2. Oxidation of Amino Acids

Experimental studies by experts show that the oxidation of leucine is enhanced during endurance exercise (its oxidation speed is directly proportional to the intensity of exercise, and the oxidation speed is 5–6 times faster than that at the maximum oxygen uptake). But whether it increases the oxidation of all amino acids remains to be proven. The intermediate metabolism of certain amino acids produces metabolites of the triolic acid cycle, which is good for muscle metabolism during exercise because it increases the oxidation capacity of the trialic acid cycle to the ethylene glycol produced by glucose and free fatty acids. In addition, metabolites of these amino acids are converted to pyruvates by phosphoenol spindle kinase and pyruvate kinase. Increased pyruvate production can lead to increased amino acid oxidation during exercise. The oxidation of amino acids is an important process of the human body. Human life is inseparable from oxygen. Oxygen is an important part of the blood.

RETRACTED

#### 2.6.3. Glucogenesis

Sugar is also an important part of the human body; exercise can consume an amount of sugar in the human body, but too much exercise can consume too much sugar, promote human hypoglycemia, and can seriously cause death. Glycosylation of amino acids is increased during exercise. It has been proved that the internal organs' absorption of gluconeoplasms is enhanced during exercise and is proportional to the intensity and duration of exercise. The gluconeogenesis process is a potentially important way to utilize amino acids because it facilitates glucose supplementation and thus prevents hypoglycemia during exercise.

In a word, a man's life is associated with many elements, but the protein is an important element; the human body needs a certain amount of protein a day to maintain body balance; athletes requirements according to the actual situation have effects on protein metabolism of human movement; athletes must have a reasonable intake of protein throughout the day to ensure normal training, which is a key factor in improving athletes' performance.

### 2.7. Current Situation of Physical Training of Aerobics Athletes in Chinese Colleges and Universities

#### 2.7.1. Lack of Basic Training

Looking at the present, for the aerobics athletes in our country's universities, although they are aerobics athletes, they are not completely the professional first-line members of the aerobics; their aerobics basis and physical health status are not very ideal, and there is also relatively a lack in the physical basic training. As far as the aerobics competition is concerned, the movement is more difficult. If the athletes feel weak in the second half of the competition, this must be caused by the lack of physical energy reserves of the athletes themselves. Then the coordination of movements may be reduced, and the endurance has a downward trend, which will have a great impact on the range, precision, and difficulty of some movements.

#### 2.7.2. The Combination of Physical Training and Technical Training Is Not Close Enough

During the daily training of aerobics athletes, the coaches only pay attention to whether the athletes have difficult movements but ignore the endurance level of the athletes. In this way, the athletes will spend more time and energy on the training of difficult movements but ignore the training of their own physical strength. For an excellent aerobics athlete, physical training and professional technical training are linked together and are inseparable; for athletes to get good results, skills and tactics training and physical training are essential.

RETRACTED

#### 2.7.3. Single Training Content and Lack of Diversity

Chinese aerobics athletes only pay attention to the physical fitness training, such as sensitivity, flexibility, and coordination. If this single-training method is used for a long time, it will cause the separation of technical training and physical training and will eventually affect the performance. However, if, contrary to what has been mentioned above, too much attention is paid to the ability of calisthenics and too little attention is paid to physical training, the same athlete's physique will rapidly decline and ultimately fail to achieve satisfactory results.

### 2.8. Single-Molecule Detection Method of Protein

Laser-induced fluorescence method refers to irradiating a sample with a laser and then detecting the fluorescence reflection of the sample. It has the advantages of high sensitivity and good selectivity. The chemiluminescence method will detect the chemiluminescence intensity of the sample to show its concentration. It has the advantages of high sensitivity, simple instrumentation, and fast analysis speed. The disadvantages are serious interference and poor photoselectivity.

Biomechanics tools mainly include optical tweezers, magnetic tweezers, and atomic force microscopes.

1. The optical tweezers method uses a focused laser beam to generate radiation pressure to form an optical trap and realizes molecular manipulation by applying force to the particles in the trap. The schematic diagram is shown in Figure 2.
2. The magnetic tweezers method observes and analyzes the movement of sample molecules by applying force to magnetized beads in a gradient magnetic field. The schematic diagram is shown in Figure 3.
3. The atomic force microscopy method investigates the surface structure and properties of sample molecules by detecting the interatomic interaction force between the sample surface and a miniature force-sensitive element. Using the optical detection method or the tunnel current detection method, the position change of the microcantilever corresponding to each scanning point can be measured, so that the information of the surface topography of the sample can be obtained. The schematic diagram is shown in Figure 4.

RETRACTED

This section studies the influence of electrolyte solution pH on protein translocation events in pores. The experiment uses BSA molecules as the research object. Bovine serum albumin (BSA), also known as the fifth component, is a globulin in bovine serum. Fitting the curve by the function of molecular time distribution, it can be seen that as the pH of the solution increases, the molecular penetration speed increases accordingly, and the greater the pH of the solution is, the more obvious the molecular penetration speed rises.

Figures 5(a) and 5(b) show the distribution diagram transit time of BSA molecules in two salt solutions with different pH = 6/8/10. It can be found that the via time of BSA molecules increases with the pH of the solution. However, the passage times in the solutions with pH equal to 6 and 8 are similar. The passage time of the latter is slightly shorter than that of the former. The passage time in the solution of pH 10 is significantly better than that in the first two solutions.

## 3. Protein Metabolism and Requirement of Athletes during Training

### 3.1. Collection and Processing of Test Samples

In this study, venous blood was collected from the athletes on Monday morning after taking the nutrition for 0, 3, 5, and 7 weeks for a total of 4 times for 7 weeks. The application of physical or chemical methods to remove or inhibit certain coagulation factors in the blood and prevent blood coagulation is called anticoagulation. The subjects prepared EDTA anticoagulation and ordinary vacuum blood collection vessels. 1 ml whole blood was extracted with the EDTA tube, and then 4 ml whole blood was extracted with the ordinary vacuum tube. The EDTA tube was immediately used for blood count in three categories.

### 3.2. Indicator Testing and Methods

The test indicators used in this study included hemoglobin, red blood cell count, hematocrit, serum iron, serum ferritin, serum transferrin, and serum transferrin receptor.

### 3.3. Determination of Serum Ferritin

adding 125I-ferritin to the ferritin standard or sample, it will generate a competitive immune response under a certain amount of specific antibody. The binding amount of ferritin to antibody is related to the ferritin content in standard or sample. After separating the binding part and the free part with immune separating agent, the radioactivity of the binding part was measured and the binding rate was calculated. The serum was provided by the Biotechnology Research Institute. The detection range was 5–320 ng.ml^−1^, and the detection limit of the cartridge was 2 ng.ml^−1^ for 2 h at 37°C. The intragroup coefficient of variation was less than 4.0%, and the intergroup coefficient of variation was less than 11.9%. The number of pulses within 1 min of the complex was counted on the sn-6958 intelligent counter.

RETRACTED

### 3.4. The Structure Design of the Plantar Pressure Sensor

The plantar pressure sensor is a portable device used to measure the interaction force between the sole of the foot and the shoe during walking. By collecting pressure change data, the pressure measuring shoe can identify and judge the human gait and provide gait for the recognition of human behavior patterns information. In order to calculate the protein consumption and requirements of athletes, an actual picture of production foot pressure measurement shoes was made, as shown in Figure 6.

The purpose of choosing sandals for the shoe body of the measuring shoes is to facilitate the mounting of other hardware and facilitate the subjects to wear in the experiment, while the addition of insoles can protect the sensor and its wiring, enhance the reliability of the system, and increase the comfort of the wearer. The pressure data collection process is shown in Figure 7.

During exercise, people have different tolerances for different parts of the body, as well as different pressure trends. The resistance value of the pressure sensor changes with the change of the pressure received. The pressure measurement circuit board needs a certain method to convert the resistance change signal into an electrical signal, thereby indirectly measuring the pressure value. Pressure sensors are distributed in various parts of the sole of the foot, and the pressure measuring board converts the resistance signal into an analog voltage signal through signal conditioning and then obtains the pressure at each point. The main physical parameters and performance indicators of the membrane pressure sensor are shown in Table 1.

This study requires the subjects to wear measurement equipment for a long period of time to perform different exercises. During the long-term exercise, the soles of the feet are stressed and the periodic motions are frequent. If the membrane pressure sensor is not properly arranged, it is easy to produce measurement points. Problems such as offset and damage to the measurement wire make the measurement data incomplete, incorrect, and incomparable at different times. The foot pressure measurement system adopts a thin film pressure sensor and a piezoresistor as the sensor probe. The varistors are arranged in a matrix. As shown in Figure 8, each thin film pressure sensor can be arranged in the pressure measuring shoe as shown in the figure, and the measuring wire can be bent and arranged to solve this problem.

RETRACTED

## 4. Study on Protein Metabolism and Requirement of Athletes during Training

### 4.1. Effect of Protein Nutrition Taken by Aerobics Athletes

1. A total of 26 female aerobics athletes were selected to participate in the experiment. Among them, 14 female athletes were randomly divided into two groups: sports group (7 with an average training period of 3.4 years) and sports + nutrition group (7 with an average training period of 4.2 years). In addition, 12 female college students (not trained) were also randomly divided into two groups: the quiet control group (6) and the quiet + nutrition group (6). The subjects took protein nutrient solution every day before breakfast. The experiment lasted for 7 weeks. The exercise group trained for 5 days a week (all days except Saturday and Sunday), 3–5 hours a day. During the experiment, no other nutritional health products were used except for normal diet and protein supplements. The changes of hemoglobin before and after the experiment are shown in Table 2 and Figure 9.
2. According to the data of the aerobics athletes in each group above, compared with week 0, the hemoglobin in the quiet + nutrition group at 5 weeks and 7 weeks increased significantly, and the increase at week 7 was larger, with a very significant difference (*P* < 0.01), and the hemoglobin level increased by 12 g/L. There was no significant increase in 2 weeks (*P* > 0.05). The hemoglobin level in the exercise group decreased significantly at 5 weeks compared with that at 0 or 3 weeks, and there was a significant difference between 5 weeks and 3 weeks (*P* < 0.05). The hemoglobin level decreased by 6 g/L at 5 weeks compared with that at 0 weeks. In the exercise + nutrition group, there was a significant increase in hemoglobin level at weeks 7, 0, or 3, and there was a very significant difference (*P* < 0.01). The hemoglobin level at week 5 was 8.17 g/L higher than that at week 0. There was no significant difference between 5 weeks and 0 weeks or 3 weeks (*P* > 0.05). The hemoglobin levels in the groups are shown in Figure 10.

### 4.2. Changes in Protein Metabolism before and after the Experiment

1. The serum transferrin receptor level in the quiet + nutrition group decreased significantly at 4 weeks, which was significantly different from that at 0 weeks and 3 weeks (*P* < 0.01) and significantly different from that at 7 weeks (*P* < 0.05). In the exercise group, the serum transferrin receptor level increased significantly at week 5, which was significantly different from that of the same group at weeks 0 and 3 (*P* < 0.05), showing that the serum transferrin receptor level at weeks 0 and 3 was significantly lower than that at week 5. There was a significant difference (*P* < 0.01) between week 5 and week 7: the level of serum transferrin receptor at week 7 was far lower than that at week 5. The changes in serum transferrin receptor (Nmol/L) in each group were compared, and specific experimental data are shown in Table 3 and Figure 11.
2. Serum transferrin receptor levels in the quiet + nutrition group at 5 weeks were significantly lower than those in the same group at 0 weeks and 3 weeks (*P* < 0.01) and those in the same group at 7 weeks (*P* < 0.05). In the exercise group, the serum transferrin receptor level increased significantly at week 5, which was significantly different from that of the same group at weeks 0 and 3 (*P* < 0.05), showing that the serum transferrin receptor level at week 0 and 3 was significantly lower than that at week 5. There was a significant difference between week 5 and week 7 (*P* < 0.01): the serum transferrin receptor level at week 7 was much lower than that at week 5. Specific data of serum transferrin receptor levels are shown in Figure 12.

RETRACTED

## 5. Conclusion

1. To participate in aerobics exercise for a long time, after heavy load exercise training, the body protein is consumed in large quantities, may accompany the phenomenon of appetite decline, and should be in the normal diet on the basis of an appropriate amount of exogenous protein supplement. For example, in order to delay the central fatigue caused by endurance exercise, in addition to scientific control of exercise load, and gradually produce biological adaptation, exogenous supplement of branched-chain amino acids can have a good recovery effect on the body. However, the supplement of branched-chain amino acids is not the more the better. Since a large dose of branched-chain amino acids can lead to the increase of blood ammonia, which may lead to hepatic encephalopathy, the supplement of branched-chain amino acids is often combined with the supplement of sugars, which can simultaneously reduce the fatty acids produced by fat decomposition and the decomposition of branched-chain amino acids.
2. According to the research in this paper, proteins are the main components that form cell structures and are biochemical catalysts and important regulators of gene expression. Any life activity of human body cannot leave the function of protein. Especially when the body is in a state of heavy exercise load and competition, the consumption of athletes increases, and the protein in the body will be catabolized. Providing high-quality protein and amino acid nutrition can supplement the function loss of athletes, enhance muscle strength, and promote hemoglobin synthesis, which is of great significance for accelerating the elimination of fatigue.
3. Amino acids and proteins are important for aerobics athletes, but a large amount of high-protein diet harms the body. First, in the process of consuming a high-protein diet, once the protein exceeds the need, it is stored in the form of fat, which directly or indirectly increases blood cholesterol, triglyceride, and LDL levels, as well as HDL and long-term consumption of high-protein foods increases the incidence of hypertension, coronary heart disease (CHD), and atherosclerosis. The results showed that the serum transferrin receptor level in the quiet + nutrition group decreased significantly after 4 weeks, which was significantly different from that of the same group at 0 weeks and 3 weeks (*P* < 0.01) and significantly different from that of the same group at 7 weeks (*P* < 0.05). In the exercise group, the serum transferrin receptor level was significantly increased at week 5, which was significantly different from that of the same group at weeks 0 and 3 (*P* < 0.05), showing that the serum transferrin receptor level at weeks 0 and 3 was significantly lower than that at week 5.
4. This article focuses on the transition from the detection of a single-protein molecule to protein interaction. First, it explores the basic physical properties of a single-protein molecule and the transport of a single-protein molecule in a confined nanopore and then develops antigen and antibody specificity. Based on the characteristics of human plantar pressure data collected by multisensor fusion technology, this paper designs a set of dynamic recognition algorithms for monitoring key gait events and monitors key protein information of athletes.

RETRACTED

## Figures and Tables

**Figure 1:** Flow chart of protein physiological function.

**Figure 2:** Working principle of mechanical tools for single-molecule detection: optical tweezers.

**Figure 3:** Working principle of mechanical tools for single-molecule detection: magnetic tweezers.

**Figure 4:** Working principle of mechanical tools for single-molecule detection: atomic force microscope.

**Figure 5:** The effect of electrolyte solution pH on protein translocation time.

**Figure 6:** Foot pressure measurement shoe.

**Figure 7:** Pressure data collection process.

**Figure 8:** Pressure sensor layout.

**Figure 9:** Comparison of hemoglobin level (G/L) among groups.

**Figure 10:** Hemoglobin levels in the groups.

**Figure 11:** Comparison of the changes of serum transferrin receptor (Nmol/L) in each group.

**Figure 12:** The specific data of serum transferrin receptor levels.

**Table 1:** Physical parameters and performance indicators.

Parameter		Unit
Thickness	0.25	mm
Length	26.2	mm
Width	15.1	mm
Induction zone diameter	10.7	mm
Measuring pressure range	0–500	N
Nonlinearity	＜±3%	-
Hysteresis	＜±4.5%	-
Response time	＜5	Us

RETRACTED

**Table 2:** hemoglobin level (G/L) among groups.

	Quiet control group (6)	Quiet + nutrition group (6)	Exercise group (7)	Exercise + nutrition group (7)
0 weeks	126.22 ± 6.45	126.23 ± 5.56	127.89 ± 4.34	122.12 ± 3.67
3 weeks	125.23 ± 11.67	133.23 ± 10.34	131.45 ± 12.89	122.89 ± 5.23
5 weeks	132.56 ± 3.18	134.33 ± 4.72	121.89 ± 3.43	126.12 ± 4.83
7 weeks	132.12 ± 4.54	135.66 ± 2.34	124.76 ± 3.36	130.22 ± 2.23

**Table 3:** Comparison of the changes of serum transferrin receptor (Nmol/L) in each group.

	Quiet control group (6)	Quiet + nutrition group (6)	Exercise group (7)	Exercise + nutrition group (7)
0 weeks	14.65 ± 0.57	14.66 ± 0.53	14.38 ± 0.56	14.33 ± 0.56
3 weeks	14.86 ± 0.42	14.54 ± 0.57	14.45 ± 0.56	14.65 ± 0.57
5 weeks	14.54 ± 0.56	13.19 ± 0.42	15.33 ± 0.54	14.33 ± 1.20
7 weeks	14.68 ± 0.55	14.52 ± 0.89	14.23 ± 0.92	14.27 ± 1.39

## Data Availability

No data were used to support this study.
